The article "Identification and Validation of a Novel Immune Infiltration-Based Diagnostic Score for Early Detection of Hepatocellular Carcinoma by Machine-Learning Strategies" was published in 2022. Journal: Gastroenterol Res Pract.

# Identification and Validation of a Novel Immune Infiltration-Based Diagnostic Score for Early Detection of Hepatocellular Carcinoma by Machine-Learning Strategies

**DOI:** 10.1155/2022/5403423

**Published:** 2022-06-14

**Authors:** Xuli Guo, Hailin Xiong, Shaoting Dong, Xiaobing Wei

**Affiliations:** Department of Oncology, Huizhou Central Hospital, Huizhou, Guangdong, China 516001

## Abstract

**Objective:**

To investigate the diagnostic gene biomarkers for hepatocellular carcinoma (HCC) and identify the immune cell infiltration characteristics in this pathology.

**Methods:**

Five gene expression datasets were obtained through Gene Expression Omnibus (GEO) portal. After batch effect removal, differentially expressed genes (DEGs) were conducted between 209 HCC and 146 control tissues and functional correlation analyses were performed. Two machine learning algorithms were used to develop diagnostic signatures. The discriminatory ability of the gene signature was measured by AUC. The expression levels and diagnostic value of the identified biomarkers in HCC were further validated in three independent external cohorts. CIBERSORT algorithm was adopted to explore the immune infiltration of HCC. A correlation analysis was carried out between these diagnostic signatures and immune cells.

**Results:**

A total of 375 DEGs were identified. GPC3, ACSM3, SPINK1, COL15A1, TP53I3, RRAGD, and CLDN10 were identified as the early diagnostic signatures of HCC and were all validated in external cohorts. The corresponding results of AUC presented excellent discriminatory ability of these feature genes. The immune cell infiltration analysis showed that multiple immune cells associated with these biomarkers may be involved in the development of HCC.

**Conclusion:**

This study indicates that GPC3, ACSM3, SPINK1, COL15A1, TP53I3, RRAGD, and CLDN10 are potential biomarkers associated with immune infiltration in HCC. Combining these genes can be used for early detection of HCC and evaluating immune cell infiltration. Further studies are needed to explore their roles underlying the occurrence of HCC.

## 1. Introduction

Hepatocellular carcinoma (HCC) is a highly aggressive malignant solid tumors and remains the major cause of cancer death across the world [1]. The development of HCC is closely associated with the infection of hepatitis B virus (HBV) and/or hepatitis C virus (HCV) [2]. There are multiple therapy strategies for various clinical characteristics of HCC. Hepatectomy, transplantation, ablation, immunotherapy, transarterial chemoembolization, and chemotherapy have been indicated to yield survival benefits [3, 4]. Among these, surgical resection can only be conducted in early-stage HCC patients. However, its mortality is still high, which largely due to early-stage tumors symptoms which are typically asymptomatic and limited treatments for individuals with advanced HCC [5]. The high morbidity and mortality rates make early screening and diagnosis of HCC even more important. The optimal curative therapy strategies for early HCC individuals include surgical resection and liver transplantation, and individuals who finished those treatments generally show a favorable outcome, with a five-year overall survival (OS) rate between 60% and 80% [6]. From a clinical perspective, improving early screening for HCC will provide the patients more opportunity for curative treatment. Thus, developing a stable and precise model for the diagnosis of individuals with early HCC will present a considerable influence on clinical outcomes. Presently, application of ultrasonography as well as serum *α*-fetoprotein (AFP) is a commonly noninvasive approach for HCC supervision. However, the sensitivity and specificity for early-stage HCC diagnosing is unsatisfactory [7]. Thus, identification of reliable and robust diagnostic biomarkers is urgent for HCC treatment.

With the increasing development in genome-sequencing technologies as well as bioinformatic algorithms, numerous molecular signatures and genetic biomarkers have been developed to enhance the diagnosis and prognosis prediction in individuals with HCC [8–10]. Recently, immunotherapy has presented promising findings [11]. Tumor-infiltrating immune cells (TIICs) are involved in the prognosis and treatment of multiple cancer types, including HCC [12–14]. However, diagnostic gene biomarkers associated with immune cell infiltration in HCC were still limited. Thus, it is still a great need to identify novel gene biomarkers for the diagnosis of HCC, especially for early-stage HCC, in clinical practice. Machine learning (ML) belongs to a subset of artificial intelligence that is widely used to solve prediction problems in human diseases by providing the machine the ability to learn from data without giving specific instructions [15, 16].

Therefore, in this study, we downloaded multiple large-scale datasets diagnosed with HCC from the GEO portal and merged into a discovery cohort after batch effect was removed. After performing differentially expressed gene (DEG) analysis, ML algorithms, including support vector machine-recursive feature elimination (SVM-RFE) and LASSO, were applied to screen candidate diagnostic genes between HCC and controls. The shared genes identified by the two methods were validated in three external validation cohorts and were used to construct the diagnostic score for early-stage HCC screening using a logistic regression method. Then, the putative abundance of immune cell subtypes via CIBERSORT algorithm was calculated. Further, the association between the gene markers and infiltrating immune cells was explored to present a reference for future research in HCC.

## 2. Materials and Methods

### 2.1. HCC Datasets

We searched and downloaded five HCC microarray expression profile datasets (GSE121248, GSE45267, GSE65372, GSE51401, and GSE14520-GPL571) from the GEO portal (http://www.ncbi.nlm.nih.gov/geo) for DEG analysis, which is a public functional genomics data repository. The characteristics of the multiple cohorts utilized in the study are presented in Table 1. GSE14520-GPL3921 cohort contained 225 HCC samples and 220 controls; gene expression data was used for external validation of the diagnostic score. Gene expression matrix of 374 HCC tissues and 50 control tissues collected from The Cancer Genome Atlas (TCGA) was used for another external validation. To yield robust diagnostic performance, the Japan Project from International Cancer Genome Consortium (ICGC-LIRI-JP) collected the RNA-Seq data of 243 HCC patients and 202 controls which was used as the third external validation cohort. Next, the probes' ID in every cohort was annotated and transformed into gene symbols according to platform annotation documents, and the probes falling to match any gene symbols were excluded. If multiple probes match to a same gene symbol, average value was used value. The gene expression files of the five datasets (GSE121248, GSE45267, GSE65372, GSE51401, and GSE14520-GPL571) were merged into a discovery cohort for subsequent analysis. The batch effects between different datasets were corrected by the R package “SVA” containing the “Combat” function [17].

### 2.2. DEG Identification

Five datasets were combined, and batch effects were eliminated by using the “Combat” algorithm. Then, these datasets were merged into a discovery cohort. There are 209 patients with HCC and 146 normal individuals in the cohort. The present study analyzed differentially expressed gene (DEG) by the “limma” R package via the comparison of the expression matrixes of HCC and control samples. The volcano plot was plotted to show the DEGs, which with thresholds of adjusted *P* < 0.05 and ∣log_2_ FC | >1 being statistically significant.

### 2.3. Functional Correlation Analysis

Gene Ontology (GO) enrichment was conducted and visualized using the “ClusterProfiler” R packages. Disease Ontology (DO) enrichment was implemented via the “ClusterProfiler” and DOSE packages [18, 19]. Gene set enrichment analysis (GSEA) was performed to seek the foremost regulated pathways and functional terms between the HCC and normal samples [20]. The “c2.cp.kegg.v7.0.symbols.gmt” was adopted as the reference gene set. The cutoff point of significance was deemed as notably enriched if a *P* < 0.05 as well as false discovery rate < 0.025.

### 2.4. Identification and Validation of Candidate Biomarkers

To construct a gene-based diagnostic score using the discovery cohort, two machine learning algorithms were selected to perform the disease status predictions. A LASSO-based algorithm, which is a regression analysis algorithm, was used for data dimensionality reduction. LASSO runs a covariate selection, which contributes to the prediction accuracy as well as the interpretability through regularization. LASSO was implemented with the “glmnet” R package to investigate the variables notably related to the discrimination of HCC and controls [21]. SVM is a supervised machine learning classification algorithm that has been commonly utilized for disease classification through predicting the extent of an individual belonging to a specific class [22]. To identify the set of genes with highest discriminative power, SVM-RFE was used to choose the suitable feature genes. The intersection genes identified by the two ML procedures were used as candidate biomarkers, and the expression values of these genes were additional confirmed in three independent external datasets.

### 2.5. Feature Gene Biomarker Selection and Diagnostic Score Construction

The validated biomarkers were used for model construction. The gene-based diagnostic score was developed via logistic regression model analysis in the discovery cohort using the following formula: diagnostic score = (*β*_1_∗Expgene_1_) + (*β*_2_∗of Expgene_2_) + ⋯+(*β*n∗Expgene_n_). The predictive significance of the diagnostic score was measured using receiver operating curve (ROC) analysis. The diagnostic scores in three external cohorts were calculated using the same formula, respectively. ROC curve was generated based on the gene expression value from HCC and normal tissues in the discovery cohort and three validation cohorts. The AUC was adopted to measure the diagnostic efficiency in separating HCC from normal samples and further verified in the validation cohorts. Moreover, the effectiveness of the diagnostic score in identifying early stage of HCC individuals (stage I) from control ones was additionally quantified in three validation cohorts via the AUCs.

### 2.6. Analysis of Immune Cell Infiltration

Infiltrating immune cells derived from the gene expression matrix in the discovery cohort in HCC were calculated by the CIBERSORT algorithm (https://cibersortx.stanford.edu/). To infer the relative abundance of infiltrating immune cells, a reference set with 22 sorted kinds of immune cell subtypes (LM22) with 1,000 permutations was adapted [23]. The R package “corrplot” was used to analyze the correlation analysis and visualize the 22 kinds of infiltrating immune cells. The “vioplot” package in R was adapted to plot violin plots and visualize the differences of immune cell infiltration between the HCC and normal tissues.

### 2.7. Investigating the Link between Selected Biomarkers and Infiltrating Immune Cells

We used CIBERSORT in R language to analyze the differences in the infiltration of 22 immune cells between the HCC and normal tissues. Spearman's rank correlation analysis was adapted to obtain the relationship between each diagnostic gene and immune cell infiltration and was visualized with “ggplot2” package.

### 2.8. Statistical Analysis

The LASSO regression analysis was implemented using the “glmnet” R package, and the SVM algorithm was carried out using the “e1071” R package. ROC curve analysis was performed to quantify the diagnostic efficacy of the diagnostic score. All statistical analyses were performed using R software (version 3.6.1), and a *P* < 0.05 was deemed statistically significant.

## 3. Results

### 3.1. Screening of Predictive Genes in HCC

DEGs were performed between 146 normal individuals and 209 patients with HCC in the discovery cohort after eliminating the batch effects (Figure 1(a)). Initially, 375 DEGs were acquired, which included 130 significantly upregulated genes and 245 significantly downregulated genes (Figure 1(b)).

### 3.2. Functional Enrichment Analysis of DEGs

The GO and KEGG analysis results show that DEGs are significantly enriched in cellular senescence, cell cycle, tubulin binding, mitotic spindle, and mitotic nuclear division (Figure 2(a)). Moreover, the functional enrichment demonstrated that diseases enriched by DEGs were generally related to non-small-cell lung carcinoma, liver cirrhosis, kidney cancer, bile duct adenocarcinoma, renal carcinoma, and breast carcinoma (Figure 2(b)). The GSEA results revealed that changed genes were enriched in several common pathways that are mainly involved in DNA replication, mismatch repair, proteasome, pyrimidine metabolism, and progesterone-mediated oocyte maturation (Figure 2(c)). These findings strongly suggest that cell cycle and cancer-related pathways play an essential role in the pathogenesis of HCC.

### 3.3. Development and Confirmation of an Immune-Related Diagnostic Gene Biomarker-Based Diagnostic Score

We performed two different bioinformatic algorithms to screen the potential biomarkers of HCC. By using the LASSO regression algorithm, DEGs were narrowed down to 29 variables as diagnostic biomarkers for HCC (Figure 3(a)). By using the SVM-RFE algorithm, we identified a subset of 40 genes among the DEGs (Figure 3(b)). The 8 overlapping feature genes (GPC3, ACSM3, SPINK1, COL15A1, TP53I3, RRAGD, CLDN10, and GPR88) were finally identified (Figure 3(c)). Moreover, in order to yield precise and reliable gene expression results, the GSE14520-GPL3921 dataset, ICGC, and TCGA-HILC cohorts were adapted to check the expression values of the 8 genes. Finally, the expression values of GPC3, ACSM3, SPINK1, COL15A1, TP53I3, RRAGD, and CLDN10 in HCC samples were particularly lower than individuals in the control cohort (Figures 4(a)–4(c); all *P* < 0.05), while the expression values of GPR88 in HCC samples were not greatly higher than individuals in the control group in GSE14520-GPL3921 dataset and ICGC (*P* > 0.05). Thus, the seven selected biomarkers were adapted to construct a diagnostic score via a logistic regression procedure. After obtaining the coefficients via multivariate logistic regression algorithm, the diagnostic score was established. Diagnostic score = (0.6325∗GPC3) + (−0.9191∗ACSM3) + (0.2633∗SPINK1) + (0.7349∗COL15A1) + (0.8170∗TP53I3) + (0.4756∗RRAGD) + (−0.8263∗CLDN10). Therefore, the diagnostic scores in four cohorts were obtained, respectively.

### 3.4. Diagnostic Effectiveness of the Diagnostic Score in HCC

We further quantified the discrimination ability by the area under a ROC curve (AUC). As demonstrated in Figure 5(a), the diagnostic capability of the seven genes in separating HCC from the normal tissues presented an excellent diagnostic performance, with all AUCs > 0.8. Considering the discriminatory ability of the diagnostic score, ROC curve analysis was performed. The AUC was 0.980 (95%CI = 0.960 − 0.990), demonstrating a high prediction efficacy of the diagnostic score gene signature for HCC. The robustness of the seven-gene diagnostic score was further confirmed in three validation cohorts for predicting diagnosis in individuals with HCC with an AUC of 0.962 in GSE14520 validation cohort (Figure 5(b)), AUC of 0.963 in ICGC cohort (Figure 5(c)), and AUC of 0.942 in TCGA-HILC cohort (Figure 5(d)), suggesting that the identified gene biomarkers had a high and strong diagnostic ability.

Additionally, we further calculated the diagnostic role of the diagnostic score gene signature for HCC at early stage (stage I). The detailed stage information was available in three validation cohorts. Surprisingly, the diagnostic score displayed high discriminability for early-stage HCC in the GSE14520 validation cohort (HCC-stage I vs. non-HCC, AUC = 0.955, Figure 6(a)), ICGC cohort (HCC-stage I vs. non-HCC, AUC = 0.952, Figure 6(b)), and TCGA-HILC cohort (HCC-stage I vs. non-HCC, AUC = 0.944, Figure 6(c)). These results demonstrate that the selected gene biomarkers presented a high diagnostic power for the early diagnosis of HCC.

### 3.5. Investigation of Immune Cell Infiltration

We explored the composition of immune cells in HCC cases and healthy controls using the CIBERSORT algorithm. The abundance of 22 immune cells in HCC and control samples was shown using a bar plot (Figure 7(a)). The proportions of CD8^+^ T cell (*P* = 0.004), resting memory CD4^+^ T cells (*P* = 0.006), gamma delta T cells (*P* < 0.001), resting NK cell (*P* = 0.001), monocytes (*P* = 0.004), M2 macrophages (*P* = 0.021), and neutrophils (*P* < 0.001) in HCC were significantly lower than in healthy controls (Figure 7(b)). However, the proportion of regulatory T cells (*P* < 0.001), activated NK cell (*P* < 0.001), M0 macrophages (*P* < 0.001), resting dendritic cell (*P* < 0.001), and activated mast cell in HCC was significantly higher than that in healthy controls (Figure 7(b)).

### 3.6. Association between the Seven Gene and Infiltrating Immune Cells

As exhibited in Figure 8, CLDN10 was positively associated with naive CD4^+^ T cells (*r* = 0.132, *P* = 0.049), CD8^+^ T cells (*r* = 0.147, *P* = 0.003), neutrophils (*r* = 0.149, *P* = 0.025), and gamma delta T cells (*r* = 0.246, *P* = 0.0002) and negatively correlated with M0 macrophages (*r* = −0.366, *P* < 0.001), activated mast cells (*r* = −0.212, *P* = 0.001), regulatory T cells (*r* = −0.199, *P* = 0.003), and activated NK cells (*r* = −0.137, *P* = 0.042). GPC3 was positively correlated with regulatory T cells (*r* = 0.145, *P* = 0.031), activated memory CD4^+^ T cells (*r* = 0.151, *P* = 0.025), activated NK cells (*r* = 0.208, *P* = 0.002), and M0 macrophages (*r* = 0.487, *P* < 0.001) and negatively correlated with resting NK cells (*r* = −0.259, *P* < 0.001), M2 macrophages (*r* = −0.252, *P* = 0.0001), monocytes (*r* = −0.248, *P* = 0.0001), gamma delta T cells (*r* = −0.225, *P* = 0.0007), and neutrophils (*r* = −0.221, *P* = 0.0009). ACSM3 was positively correlated with CD8^+^T cells (*r* = 0.136, *P* = 0.043), resting memory CD4^+^ T cells (*r* = 0.156, *P* = 0.020), M1 macrophages (*r* = 0.204, *P* = 0.002), resting NK cells (*r* = 0.259, *P* < 0.001), and delta gamma T cells (*r* = 0.321, *P* < 0.001) and negatively correlated with naive CD4^+^ T cells (*r* = −0.144, *P* = 0.032), plasma cells (*r* = −0.151, *P* = 0.024), activated NK cells (*r* = −0.221, *P* = 0.001), regulatory T cells (*r* = −0.267, *P* < 0.001), and M0 macrophages (*r* = −0.385, *P* < 0.001). SPINK1 was positively correlated with M0 macrophages (*r* = 0.346, *P* < 0.001), activated NK cells (*r* = 0.205, *P* = 0.002), and regulatory T cells (*r* = 0.163, *P* = 0.015) and negatively correlated with monocytes (*r* = −0.144, *P* = 0.033), resting NK cells (*r* = −0.162, *P* = 0.016), CD8^+^ T cells (*r* = −0.245, *P* = 0.0001), and delta gamma T cells (*r* = −0.258, *P* = 0.0001). COL15A1 was positively correlated with regulatory T cells (*r* = 0.134, *P* = 0.047), resting dendritic cells (*r* = 0.175, *P* = 0.009), activated NK cells (*r* = 0.175, *P* = 0.009), and M0 macrophages (*r* = 0.415, *P* < 0.001) and negatively correlated with delta gamma T cells (*r* = −0.307, *P* < 0.001), resting NK cells (*r* = −0.305, *P* < 0.001), neutrophils (*r* = −0.261, *P* < 0.001), and CD8^+^ T cells (*r* = −0.243, *P* < 0.001). TP53I3 was positively correlated with M1 macrophages (*r* = 0.161, *P* = 0.016), resting dendritic cells (*r* = 0.189, *P* = 0.005), regulatory T cells (*r* = 0.226, *P* < 0.001), activated NK cells (*r* = 0.315, *P* < 0.001), and M0 macrophages (*r* = 0.424, *P* < 0.001) and negatively correlated with delta gamma T cells (*r* = −0.361, *P* < 0.001), resting NK cells (*r* = −0.323, *P* < 0.001), CD8^+^ T cells (*r* = −0.258, *P* < 0.001), resting memory CD4^+^ T cells (*r* = −0.221, *P* < 0.001), neutrophils (*r* = −0.217, *P* = 0.001), and activated dendritic cells (*r* = −0.170, *P* = 0.011). RRAGD was positively correlated with M0 macrophages (*r* = 0.439, *P* < 0.0001), activated NK cells (*r* = 0.241, *P* < 0.001), regulatory T cells (r = 0.202, *P* = 0.003), plasma cells (*r* = 0.161, *P* = 0.017), and activated mast cells (*r* = 0.146, *P* = 0.030) and negatively correlated with neutrophils (*r* = −0.148, *P* = 0.028), resting NK cells (*r* = −0.188, *P* = 0.005), resting memory CD4^+^ T cells (*r* = −0.211, *P* = 0.002), CD8^+^ T cells (*r* = −0.301, *P* < 0.001), and delta gamma T cells (*r* = −0.472, *P* < 0.001).

## 4. Discussion

In recent years, numerous reports have endeavored to demonstrate the pathogenesis and pathomechanism of HCC. Despite that huge development on surgical treatment and drug therapy has been acquired, the outcome of HCC is still unsatisfactory. Without powerful diagnosis approach on the early stage often results in poor progression of HCC. Therefore, developing stable prognostic biomarkers that reveal the biological progression of the HCC will be vital for its prevention and treatment.

In the current study, we constructed an integrated bioinformatic analysis to determine diagnostic genes that are involved in immune cell infiltration in individuals with HCC. Seven potential immune-related diagnostic gene biomarkers (GPC3, ACSM3, SPINK1, COL15A1, TP53I3, RRAGD, and CLDN10) were identified for HCC using two machine learning algorithms. In addition, these candidate biomarkers were strongly related to multiple immune cells. These feature genes and immune cells may offer new promising early diagnostic and immunotherapeutic strategies for HCC. The diseases enriched by DEGs were observed to be mainly associated with cancer-related pathways. GO and KEGG analysis results show that DEGs are significantly enriched in cell cycle, tubulin binding, mitotic spindle, and mitotic nuclear division, highly associated with HCC oncological diseases, suggesting cell cycle exerts a strong influence on the development and homeostasis of HCC. Deregulated cell cycle process is a hallmark of malignancy, and targeting CDKs to inhibit cell proliferation has been approved as a helpful anticancer therapy [24] [25]. Abnormalities in cell cycle mechanisms often accompany HCC carcinogenesis. Based on these findings, the results in our study may present potential targets for the therapy of HCC.

HCC is a highly heterogeneous malignant solid tumor. Cells of the immune system are indispensable regulators for tumor microenvironment (TME) homeostasis. The TME comprises the stromal as well as immune cells which interact with or infiltrate a particular cancer [26]. Among the TME, immune cells are the key factors of tumor progression. At the same time, immunotherapy is a promising tumor-killing method. The degree of infiltration of immune cells can reflect the response of HCC cells to immunotherapy, as well as different prognoses. However, despite the development of immunotherapy for HCC, the results have not been satisfactory. Immune cell infiltration and distribution are highly heterogeneous and complex, and the search for factors driving immune infiltration or key biomarkers is crucial to reveal this heterogeneity. In HCC, TME is immunosuppressive and contributes to immune tolerance and evasion via multiple processes, boosting cancer proliferation, invasion, and metastasis [26]. Presently, increasing investigations have illustrated that the effector of CD8+, regulatory T cells, CD4^+^ cells, and dendritic cells could affect the effectiveness of immune checkpoint inhibitors [27, 28]. In this present study, by using CIBERSOTR algorithm, a great diversity of the infiltrated immune cells was found to be participating in the process of HCC. In detail, regulatory T cell, activated NK cells, M0 macrophages, resting dendritic cell, and activated mast cell were decreased in HCC cohort. This evidence is in general agreement with our results that multiple immune cells are associated with these biomarkers, suggesting that a substantial amount of immune cell is involved in HCC. Therefore, identifying potential gene biomarkers correlated with immune cell infiltration for HCC will contribute to its diagnosis and treatment.

GPC3, ACSM3, SPINK1, COL15A1, TP53I3, RRAGD, and CLDN10 were identified as potential new immune-related diagnostic biomarkers with high diagnostic value, which may serve as ideal biomarkers for the diagnosis of HCC, as well as for the early stage of HCC. In recent years, machine learning has been applied to various fields of biomedicine. Compared with most traditional statistical methods, the advantage of machine learning is that it can identify potential rules through massive data learning. Machine learning algorithms have been applied to identify cancer prognostic characteristic genes and tumor classification [29]. Machine learning is a crucial discipline of artificial intelligence, utilizes procedures that identify patterns within existing data, and trains itself to perform predictions on other data [30]. Glypican-3 (GPC3) belongs to a member of the glypican family, which has been utilized as a potential diagnostic biomarker for HCC owning to its preferential expression in HCC [31]. GPC3 was highly expressed in HCC samples than in benign liver lesions, which may play an important role in HCC diagnosis than alpha-fetoprotein (AFP) [32]. ACSM3 was downregulated in HCC, and individuals with little expression of ACSM3 presented miserable prognosis. High expression of ACSM3 weakened migration and invasion of HCC cells *in vitro* and *in vivo* as well as downregulated the phosphorylation of WNK1 and AKT [33]. SPINK1 is highly expressed and contributes to cancer progress in multiple cancers, including HCC. It has been proved that SPINK1 increased proliferation and promoted migration and invasion capability of HCC cell lines [34]. CLDN10 expressed highly in HCC cells, and growing evidence demonstrates that CLDN10 is functionally involved in HCC invasion and is a possible target for HCC therapy [35]. Furthermore, knockdown of CLDN10 by siRNA reduced HCC cell migration [36]. COL15A1 is a novel atherosclerosis gene that is involved in vascular smooth muscle cell phenotype, which is regulated by epigenetic state in passaged cells and located in atherosclerotic tissue [37]. However, the diagnostic and prognostic role of COL15A1 in HCC remains unknown. TP53I3, one of the p53-induced genes, is an oxidoreductase-like protein that is transcriptionally activated by the tumor suppressor TP53 and involved in TP53-mediated apoptosis as well as DNA damage response [38]. As we know, TP53 mutation is one of the common alterations in multiple cancers, including HCC. Mutations in the TP53 gene could yield genetic instability and result in cancer progression [39]. RRAGD encodes a small Rag guanosine triphosphatase, which is an important component of the nutrient-sensing pathway that activates mTOR signaling [40]. The relationship between mTOR signaling pathway and the pathogenesis of HCC has been widely confirmed previously [41, 42].

To deeply evaluate the diagnostic performance of the model, this signature was sufficiently validated and evaluated in multiple different external validation datasets, revealing the robustness and reliability of the diagnostic score. Despite the use of bioinformatics and machine learning algorithms in our study and the discovery of the diagnostic value of key genes in HCC patients, several limitations still exist in present study. First, the findings concluded from bioinformatics analysis need RT-PCR in clinical tissues to additional verify. Besides, most of the identified genes need *in vitro* and *in vivo* validation experiments in HCC, and further evidence provided by a well-designed study is required.

## 5. Conclusion

In summary, we identified GPC3, ACSM3, SPINK1, COL15A1, TP53I3, RRAGD, and CLDN10 as diagnostic immune-related biomarkers with potential clinical utility, which might have the ability to accurately early diagnosis of HCC, enable earlier access to intervention, and improve the clinical outcomes. Moreover, multiple immune cells may be involved in the occurrence and development of HCC and could be used as potential targets for future immunotherapy in patients with HCC that warrant further investigations.

## Figures and Tables

**Figure 1:** Differentially expressed genes (DEGs) identified between HCC and control samples. (a) Heatmap of DEG distribution and (b) volcano plots of DEG distribution.

**Figure 2:** Functional enrichment analysis. (a) GO and KEGG functional enrichment analyses of the DEGs. (b) Disease Ontology enrichment analysis of the DEGs between HCC and control samples. (c) Enriched gene set enrichment analysis (GSEA) terms between HCC and controls.

**Figure 3:** Screening for potential diagnostic gene biomarkers of HCC by two machine learning strategies. (a) Screening diagnostic gene biomarkers using the least absolute shrinkage and selection operator (LASSO). (b) The optimal gene biomarker selection via support vector machine-recursive feature elimination (SVM-RFE) algorithm. (c) Venn diagram displaying eight diagnostic biomarkers shared by LASSO and SVM-RFE algorithms.

**Figure 4:** Verification of the expression levels of selected diagnostic gene markers in three validation cohorts. (a) GSE14520-GPL3921 cohort. (b) ICGC-LIRI-JP cohort. (c) TCGA cohort.

**Figure 5:** The ROC curve of the discrimination ability of the seven identified diagnostic gene biomarkers in different cohorts. (a) The discovery cohort. (b) GSE14520-GPL3921 cohort. (c) ICGC-LIRI-JP cohort. (d) The TCGA cohort.

**Figure 6:** The ROC curve of the discrimination ability of the seven identified diagnostic gene biomarkers for early-stage HCC in cohorts. (a) GSE14520-GPL3921 cohort. (b) ICGC-LIRI-JP cohort. (c) The TCGA cohort.

**Figure 7:** The view of immune infiltration between HCC and controls. (a) Violin diagram of the proportion of 20 types of immune cells between HCC and normal controls. (b) The difference of immune infiltration between HCC and normal controls.

**Figure 8:** Correlation analyses between diagnostic gene biomarkers and infiltrating immune cells in HCC. Correlation between GPC3, ACSM3, SPINK1, COL15A1, TP53I3, RRAGD, CLDN10, and infiltrating immune cells. The size of the dots represents the strength of the correlation between feature genes and immune cells; the larger the dots, the stronger the correlation.

**Table 1:** Details of the multiple datasets included in this study.

Datasets	Platform	Sample size (tumor/control)	Application
GSE121248	GPL570 [HG-U133_Plus_2] Affymetrix Human Genome U133 Plus 2.0 Array	107 (70/37)	Identification of DEGs

GSE45267	GPL570 [HG-U133_Plus_2] Affymetrix Human Genome U133 Plus 2.0 Array	87 (48/39)	Identification of DEGs

GSE65372	GPL14951 Illumina HumanHT-12 WG-DASL V4.0 R2 expression beadchip	54 (39/15)	Identification of DEGs

GSE51401	GPL570 [HG-U133_Plus_2] Affymetrix Human Genome U133 Plus 2.0 Array	64 (30/34)	Identification of DEGs

GSE14520	GPL571 [HG-U133A_2] Affymetrix Human Genome U133A 2.0 Array	43 (22/21)	Identification of DEGs

GSE14520	GPL3921 [HT_HG-U133A] Affymetrix HT Human Genome U133A Array	445 (225/220)	Validation of DEGs

ICGC-JP cohort		445 (243/202)	Validation of DEGs

TCGA-HILC		424 (374/50)	Validation of DEGs

## Data Availability

Multiple publicly cohort data were used in the present study. The data utilized in present study are downloaded from the open GEO data database (https://www.ncbi.nlm.nih.gov/geo/; accession numbers: GSE14520, GSE45267, GSE51401, GSE65372, and GSE121248), TCGA data portal (https://portal.gdc.cancer.gov/), and ICGC data portal (https://dcc.icgc.org/).
